The article "Effect of Narrative Nursing on Family Resilience and Psychosocial Adaptation of Middle-Aged Patients with Breast Cancer" was retracted in 2023. Reasons: signs of a paper mill; suspected computer-generated content; unreliable results or conclusions; lack of ethics approval or compliance.

# Effect of Narrative Nursing on Family Resilience and Psychosocial Adaptation of Middle-Aged Patients with Breast Cancer

**DOI:** 10.1155/2022/5499298

**Published:** 2022-09-13

**Authors:** Xiaohong Jin, Xiaoman Liu, Huiwen Xie, Jie Yu, Dongmei Gu

**Affiliations:** Department of Nursing, Affiliated Hospital of Nantong University, Nantong, China

## Abstract

Patients with breast cancer frequently experience psychological distress. This study aimed to investigate the effect of narrative nursing on middle-aged patients with breast cancer. In all, 82 patients with breast cancer admitted to the Affiliated Hospital of Nantong University were divided into two groups, namely, the observation group and the control group, by simple random sampling, with 41 cases in each group. The patients in both groups were treated with breast cancer surgery. Additionally, the control group received routine nursing, whereas the observation group received narrative nursing based on the control group. After 8 weeks of nursing, the SAS (self-rating anxiety scale) and SDS (self-rating depression scale) scores in the observation group were lower than those in the control group (*P* < 0.01). At the same time, the result of family hardiness showed that the patients with narrative nursing performed better in commitment, challenge, and control (*P* < 0.01). In conclusion, narrative nursing can alleviate the postoperative shame and negative emotions of patients with breast cancer and improve their quality of life.

## 1. Introduction

Owing to the high incidence rate and high mortality of breast cancer, it is currently the largest malignant tumor that endangers women's health worldwide [1]. According to the latest global cancer data, breast cancer has increased by 2.26 million, surpassing lung cancer for the first time and becoming the most common cancer worldwide [2]. With the development of early diagnosis and treatment technology, the survival rate and survival time of patients with breast cancer have increased yearly [3]. Surgery can remove the breast tissue invaded by cancer cells. Postoperative chemotherapy can consolidate the therapeutic effects, reduce the recurrence rate of cancer after surgery, and prolong the survival time of patients [4]. Patients need long-term survival with cancer, and their psychosocial adaptability directly determines the quality of life with cancer [5]. Living with a chronic disease has a profound impact on the physical, psychological, and social quality of life [6]. Patients with breast cancer often have a series of psychosocial problems after undergoing stressful events, such as a cancer diagnosis and mastectomy. Additionally, postoperative trauma and unknown and uncertain chemotherapy aggravate the psychological pain of patients. Research shows that the detection rate of psychological distress in patients with breast cancer is 24.2%–78.2%, which affects the ability of patients to recover physical functions and cope with diseases [7].

The article "Effect of Narrative Nursing on Family Resilience and Psychosocial Adaptation of Middle-Aged Patients with Breast Cancer" was retracted in 2023. Reasons: signs of a paper mill; suspected computer-generated content; unreliable results or conclusions; lack of ethics approval or compliance.

According to the World Health Organization's criteria for age classification, middle-aged people are 45–59 years old, middle-aged women are the pillar of a family and mainstay of the unit, and work is the main source of family income. Due to diseases and treatment-related factors, many patients are forced to stop working, which will lead to a decline in the quality of life due to personal factors, such as a sense of restriction and economic factors, and thereby increase the burden of disease and the risk of suicide. Age is an important factor that affects the occurrence of negative emotions, such as anxiety and depression, in patients with breast cancer. Therefore, alleviating the negative emotional experience of middle-aged women with breast cancer is an effective way to improve treatment compliance, reduce complications, reduce mortality, prolong survival, and improve the quality of life of such patients. In terms of physiology, a study found that pressure activates the neuroendocrine-immune axis to release inflammatory mediators and immune factors, reduces the body's resistance, causes infection, accelerates aging, increases the risk of cardiovascular diseases, and weakens the monitoring role of the immune system to identify and clear malignant cells, so as to make cancer relapse and metastasize [8]. Therefore, exploring safe and effective intervention measures to reduce physical and mental stress and improve the mental state and immune function of patients with breast cancer is the key to improving their quality of life, and it is also a research hotspot in recent years. To this end, this study used narrative nursing to intervene with middle-aged patients with breast cancer and explored the relationship of narrative nursing with family resilience, psychosocial adaptation, and immune function of middle-aged women with breast cancer to further improve the quality of life of middle-aged patients with breast cancer.

## 2. Materials and Methods

### 2.1. Preparation

The team consisted of one head nurse with a psychological consultant certificate and five experienced department nurses (members of the department of mental health team). All members participate in early systematic learning, master the narrative psychological counseling technology, and meet the requirements. The members are responsible for the following contents:

1. Quality control administrator: served as the nursing backbone, engaged in nursing work for many years, engaged in psychological counseling and breast cancer nursing for many years, and participated in hospice care, narrative nursing, and other classes. By analyzing the narrative nursing record sheet and reflection diary of narrative nurses, we can correct and improve the narrative nursing method and improve the quality of nursing service.
2. Psychological nursing assistant: composed of one head nurse with a psychological consultant certificate and two department nurses (members of the department of mental health team) who were responsible for guiding narrative nurses to establish relations with patients, guide specific nursing work, and improve daily nursing work during the narrative process.
3. Narrative nursing practitioner: two nurses were responsible for the long-term work in the cancer ward and personally carried out clinical nursing based on the following criteria: have mastered the general knowledge of postoperative nursing of patients with breast cancer, the key points of postoperative rehabilitation nursing, and narrative nursing skills. Know that patients should be respected and not harmed in the narrative nursing process and should be treated with enthusiasm, humility, and love. Master the five core narrative techniques and their comprehensive application methods, get familiar with patients, establish contact with patients, and further guide and encourage patients through narration.

The article "Effect of Narrative Nursing on Family Resilience and Psychosocial Adaptation of Middle-Aged Patients with Breast Cancer" was retracted in 2023. Reasons: signs of a paper mill; suspected computer-generated content; unreliable results or conclusions; lack of ethics approval or compliance.

### 2.2. Patients, Settings, and Procedures

Eligibility requirements included age 45–59 years, cancer diagnosis at any stage, and completion of initial chemotherapy, with the ability of Chinese participants to provide informed consent and their refusal to participate in other psychosocial studies. Participants were recruited by clinicians or by research nurses in waiting rooms of clinics that were not recruiting for other psychosocial studies. Clinicians and research nurses described the study as a comparison between the two interventions described above, and they could experience the other group's intervention at the end of the study. The patients received a brochure and the informed consent form and, if interested, signed a form giving them permission to contact the first author for an informational and consenting interview. Participants were randomized in a 1 : 1 ratio after signing the consent form and completing an online baseline survey based on WeChat. Participants were not blinded to the intervention but were blinded to which intervention was the control and which was the treatment condition.

### 2.3. Negative Emotions

The self-rating depression scale (SDS) was used to evaluate the severity of depression in patients. A score of 53–62 indicates mild depression, 63–72 indicates moderate depression, and 73–100 indicates severe depression. The self-rating scale (SAS) was used to evaluate the severity of anxiety. A score of 50–59 denotes a mild case of anxiety, 60–69 points a moderate case of anxiety, and 70–100 points a severe case of anxiety.

The article "Effect of Narrative Nursing on Family Resilience and Psychosocial Adaptation of Middle-Aged Patients with Breast Cancer" was retracted in 2023. Reasons: signs of a paper mill; suspected computer-generated content; unreliable results or conclusions; lack of ethics approval or compliance.

### 2.4. Family Hardiness Index

McCubbin developed and tested the Family Hardiness Index to evaluate family hardiness. Yang Liu translated and modified this index for the Chinese context and administered it to the parents of 330 hospitalized children in 2011. The Chinese version consists of 20 items, ranging from 1 to 4 (1 = “false” and 4 = “true”), covering commitment, challenge, and control. Total scores for family hardiness, which ranged from 20–80, were calculated by summing the items in each domain. The high scores indicated high levels of family hardiness. The Cronbach's alpha value obtained for the total Chinese scale was 0.803 [9, 10].

### 2.5. Statistical Methods

The *R* language was used for data analysis. The measurement data and enumeration data were expressed as (mean ± sd) and *n* (%), respectively, and Student's *t*-tests and *χ*2 tests were used for comparison between groups, respectively. *P* < 0.05 was considered statistically significant.

## 3. Results

### 3.1. Comparing Clinical Characteristics

Of the total number of respondents, 82 patients were included. The mean age (±SD) of participants was 52.22 ± 3.94 years in the control group and 52.29 ± 4.43 in the treatment group, ranging between 45 and 59 years. No significant differences in clinical characteristics were observed between the two groups (Table 1).

### 3.2. Changes in SAS and SDS Scores

The SAS and SDS were adopted for evaluating patients' anxiety and depression before and after the intervention, respectively. According to the results, before the intervention, the two groups had similar SAS and SDS scores (both *P* > 0.05). However, after the intervention, the SAS and SDS scores of both groups decreased significantly, with lower SAS and SDS scores in the treatment group than those in the control group (both *P* < 0.001) (Table 2; Figures 1(a) and 1(b)).

### 3.3. Correlations between Family Hardiness

The average family hardiness scores were 52.76 ± 5.17 (control group) and 63.81 ± 4.03 (intervention group) for the three dimensions examined: commitment (the control group: 25.32 ± 3.12, intervention group 27.32 ± 2.16), control (the control group: 12.24 ± 2.29, intervention group 19.24 ± 2.30), and challenge (the control group: 12.24 ± 2.29, intervention group 17.24 ± 2.11) (Table 3; Figure 1(c)).

## 4. Discussion

Adaptation is a systemic reaction process covering physiological, psychological, social, cultural, and technical aspects [11]. After many stressful events, such as cancer, surgery, and chemotherapy, patients stimulate their own dynamic regulation system to constantly adapt to changes in internal and external environments. The coping process under this pressure is psychosocial adaptation. Low or poor psychosocial adaptation affects the treatment, prognosis, rehabilitation, and quality of life of patients [12]. Therefore, incorporating effective methods to improve the psychosocial adaptation of patients has been the focus of researchers.

The article "Effect of Narrative Nursing on Family Resilience and Psychosocial Adaptation of Middle-Aged Patients with Breast Cancer" was retracted in 2023. Reasons: signs of a paper mill; suspected computer-generated content; unreliable results or conclusions; lack of ethics approval or compliance.

Narrative nursing, as a humanistic nursing method, combines the spirit of narrative psychotherapy and narrative medicine and is a supplement to the connotation of humanized nursing service. It implies that, through listening and absorbing the patient's story, we can help the patient realize the meaning of reconstruction of life and disease, find the key points of nursing, and then implement nursing intervention for the patient. Different from the traditional psychology school, this model emphasizes the individual's interpretation of internal emotion, value, and meaning and pays attention to tapping their problem-solving ability and self-potential, so that they can actively solve problems and face life. It is divided into four stages, namely understanding, feedback, reflection, and witness. Understanding is the premise of narration. Feedback is a further deconstruction of the patient's problems. It uses the story of the patient or others to give back to the patient and stimulate the patient's own resources and strength. Reflection is the key to the formation of internal power, including patient reflection and nurse reflection. Through reflection, the patients recognize themselves again. Nurses further improve their nursing plan and narrative ability through reflection on narrative materials, such as narrative notes, sharing meetings, and seminars.

Narrative nursing restores the medical temperature, understands and is close to the patient, places the patient at the center, and supports and encourages the patient with the patient's story, all of which are conducive to improving the 'patient's emotion and the quality of nursing service. However, China is still in the exploratory stage of narrative nursing practice. In recent years, some scholars have applied the narrative research method to the clinical practice of tumor patients and dying patients. The results show that this method improves the overall quality of care for tumor patients, relieves the psychological pain of patients, and can innovate the nursing practice of humanistic care for tumor patients and dying patients. Therefore, the practice of narrative nursing provides new perspectives, ideas, and ways for nursing patients with breast cancer.

The article "Effect of Narrative Nursing on Family Resilience and Psychosocial Adaptation of Middle-Aged Patients with Breast Cancer" was retracted in 2023. Reasons: signs of a paper mill; suspected computer-generated content; unreliable results or conclusions; lack of ethics approval or compliance.

Because middle-aged patients with breast cancer are in their prime of life, they are unable to realize their own value and affect their lives and families due to the impact of diseases. However, there are few studies specifically targeting middle-aged patients with breast cancer. This study focused on the high incidence of middle-aged patients with breast cancer and explored the impact of narrative nursing on family resilience and psychosocial adaptation of middle-aged patients with breast cancer to further improve their quality of life. For middle-aged patients with breast cancer, narrative nursing should be used to explore the inner world of patients, enrich their psychotherapy programs, improve their family's resilience, and improve their quality of life from a new perspective, to provide personalized psychological nursing for patients with the same or similar backgrounds, and further promote narrative nursing.

## Figures and Tables

**Figure 1:** (a) Line chart of SAS trends. (b) Line chart of SDS trends. (c) Boxplot of Family Hardiness including commitment, control, and challenges.

**Table 1:** Baseline of patients.

Characteristic	Control	Treat	*P*
*n*	41	41	
Work status, *n* (%)			0.631
Not working/retirement	30 (36.6%)	27 (32.9%)	
Working	11 (13.4%)	14 (17.1%)	
Education, *n* (%)			0.790
High school or above	31 (37.8%)	33 (40.2%)	
Junior high school or below	10 (12.2%)	8 (9.8%)	
Medical insurance, *n* (%)			0.755
With	34 (41.5%)	36 (43.9%)	
Without	7 (8.5%)	5 (6.1%)	
Age, mean ± SD	52.22 ± 3.94	52.29 ± 4.43	0.937
SAS Before intervention, mean ± SD	63.95 ± 3.59	62.95 ± 4.6	0.276
SDS Before intervention, mean ± SD	62.73 ± 2.75	63.05 ± 2.52	0.588

**Table 2:** Comparison of SAS scores and SDS scores.

Group	*n*	SAS			SDS		
		Before intervention	4 weeks after intervention	8 weeks after intervention	Before intervention	4 weeks after intervention	8 weeks after intervention
control	41	63.95 ± 3.59	49.27 ± 2.31	47.68 ± 4.44	62.73 ± 2.75	55.76 ± 2.74	48.44 ± 3.54
Intervention	41	62.95 ± 4.60	47.27 ± 2.44	38.51 ± 3.55	63.05 ± 2.52	52.49 ± 2.31	39.68 ± 3.13
*P* value		*P* > 0.05	*P* < 0.01	*P* < 0.01	*P* > 0.05	*P* < 0.01	*P* < 0.01

**Table 3:** Correlation between family hardiness.

Variables	Control	Intervention	*P*
commitment	25.32 ± 3.12	27.32 ± 2.16	*P* < 0.01
control	15.20 ± 2.29	19.24 ± 2.30	*P* < 0.01
challenges	12.24 ± 2.29	17.24 ± 2.11	*P* < 0.01
Overall	52.76 ± 5.17	63.81 ± 4.03	*P* < 0.01

## Data Availability

All data have been uploaded.
